The article "Effectiveness of Augmented Reality for Lower Limb Rehabilitation: A Systematic Review" was published in 2022. Journal: Appl Bionics Biomech.

# Effectiveness of Augmented Reality for Lower Limb Rehabilitation: A Systematic Review

**DOI:** 10.1155/2022/4047845

**Published:** 2022-07-18

**Authors:** Hongbin Chang, Yang Song, Xuanzhen Cen

**Affiliations:** ^1^General Studies Teaching Department, Zhejiang Fashion Institute of Technology, Zhejiang 315211, China; ^2^Doctoral School on Safety and Security Sciences, Obuda University, Budapest 1034, Hungary; ^3^Faculty of Engineering, University of Szeged, Szeged 6720, Hungary

## Abstract

Augmented reality- (AR-) based interventions have shown potential benefits for lower limb rehabilitation. However, current literature has not revealed these benefits as a whole. The main purposes of this systematic review were to determine the efficacy of AR-based interventions on lower limb recovery of the larger population based on the current process that has been made in this regard. Relevant studies were retrieved from five electronic databases (Web of Science, PubMed, ScienceDirect, Scopus, and Cochrane Library) using “augmented reality” OR “AR” AND “lower limb” OR “lower extremity” AND “intervention” OR “treatment”. Sixteen studies that met the eligibility criteria were included in this review, and they were further grouped into three categories based on the participant types. Seven studies focused on the elderly adults, six on the stroke patients, and the last three on Parkinson patients. Based on the findings of these trials, the significant effects of AR-based interventions on lower limb rehabilitation (i.e., balance, gait, muscle, physical performance, and fall efficacy) have been initially confirmed. Favorable results were achieved at least the same as the interventions without AR except for the turning and timing in the freezing of gait of Parkinson patients. However, given the infancy of this technology in clinical practices, more robust trials with larger sample sizes and greater homogeneity in terms of devices and treatment settings are warranted for further verification.

## 1. Introduction

Nowadays, advanced technologies are becoming increasingly common as rehabilitation therapeutic tools in the healthcare setting [1–6]. Among them is virtual reality (VR), which immerses the users into the artificial environment created by the computer simulation [7, 8]. Compared to the conventional retraining techniques, VR technology is considered motivating and engaging, and it offers an artificial environment where the training environment, the difficulty level of tasks, and the feedback types could be relatively effortlessly manipulated [9]. Previous studies have found that participants were more actively engaged in the VR-based rehabilitation training than the conventional one to improve motor ability [10–12]. VR has now been incorporated into varied clinical practices such as poststroke rehabilitation, and it has shown significant effects on improving the motion functions, dynamic balance, and muscle force of both upper and lower limbs among stroke patients [13, 14]. Nevertheless, emerging evidence has concerned the safety of using VR technology in clinical practices, especially for the rehabilitation training of patients with lower limb impairments [9, 15, 16]. For example, the patients may not be able to recognize their body position when using a head-mounted display (HMD) VR device, which would further lead to unexpected physical injuries [9].

Due to the above limitations, the requirement for a safer and automatic rehabilitation training tool has accumulated. In recent years, the introduction of augmented reality (AR) into clinical applications has been proposed and verified [17–19]. AR could be a safer alternative to VR since it does not fully place the users into the simulated environment but add the fundamental elements of rehabilitation training on a real-world view [20]. In addition, compared to these interactive elements designed by VR in the virtual world, the interactive elements created by AR in the real world could induce much more embodiment to the users [18]. There are emerging studies that reported the benefit of using AR for clinical rehabilitation, and several systematic reviews have further confirmed the promising effects, especially for stroke patients [17–19, 21–23]. Despite that, no review to our knowledge has investigated whether AR-based methods are beneficial for a wide range of adults such as the elderly, stroke patients, and patients with cerebral palsy or multiple sclerosis. Moreover, since the lower limbs are directly involved in most of the daily movement, it is important to further determine if AR-based methods can help to improve the lower limb rehabilitation of these above patients.

As AR technology becomes much more accessible, AR-based treatments could be widely used not only in clinical practices but also in home settings for function rehabilitation. Therefore, this review summarized and analyzed the efficacy of AR-based interventions on lower limb recovery based on the current process that has been made in this regard, aiming to determine whether it could contribute significant benefits to the larger population and further add help to guide future utilization of AR technology.

## 2. Materials and Methods

### 2.1. Search Strategy

Five English databases including Web of Science, PubMed, ScienceDirect, Scopus, and Cochrane Library were searched independently by two authors to identify relevant studies published from the very beginning until 1 June 2022. The searching keywords include “augmented reality” OR “AR” AND “lower limb” OR “lower extremity” AND “intervention” OR “treatment”. In addition, both the reference lists of the included studies and the retrieved reviews were further searched to identify other relevant articles.

### 2.2. Eligibility Criteria

In this review, two investigators assessed the retrieved studies independently, and the third investigator would be consulted if any inclusion disagreements happened. The literature exclusion was initially conducted by screening the titles and abstracts, and then, the investigators would screen the full texts of the papers for further confirmation. The eligibility criteria were formed based on participants, experimental design, and outcomes; (1) subjects: studies that reported the effects of AR-based interventions/applications on lower limb rehabilitation of both healthy participants and patients without age limit were included; (2) experimental design: this review focused on the effectiveness of AR for lower limb rehabilitation, and therefore, any randomized controlled trials or observational studies related to this topic were all included; (3) outcomes: the study results should include variables related to lower limb rehabilitation, such as gait kinematics, muscle strength, and balance. In addition, only English original researches published on peer-reviewed journals were included in this study, while reviews, conference proceedings, and study protocols were excluded.

### 2.3. Data Extraction

The following data from included studies were further extracted and summarized by two investigators and verified by the third one: (1) author, including the name of the first author and published year; (2) study purposes; (3) participant, including the number of participants, age, gender, and physical conditions; (4) intervention, experimental design, and intervention protocols (type, frequency, time, total duration); (5) comparison and comparison protocols (type, frequency, time, total duration); and (6) outcome, the primary findings of these studies. In addition, the Mendeley Desktop Reference Management Software (Mendeley Ltd., Netherlands) was applied for organizing articles and generating citations.

## 3. Results

### 3.1. Search Results

The flow chart of the search procedure of this review is presented in Figure 1. A total of 259 papers were initially searched from the five databases. It was reduced to 11 articles after screening according to the eligibility and removing all the duplicates. Five additional papers were identified from the reference lists of these retrieved studies, which makes it in total 16 studies included in this review. Most studies compared the effects of AR interventions with the corresponding control programs, while there are also some studies that evaluated the before-after effects without any control trials. Conventional physical fitness program was normally conducted for control groups; however, some studies also offered insight from other directions, such as Tai Chi, yoga, and functional electrical stimulation. Over half of the studies were performed on elderly adults (*n* = 7), and the rest of the studies were performed on stroke patients (*n* = 6) and Parkinson patients (*n* = 3). The detailed study characteristics are summarized in Table 1, and these included studies were further grouped into three categories based on the types of participants to elaborate the acute or chronic effects of AR interventions on lower limb rehabilitation.

### 3.2. AR Rehabilitation Systems

Most of the AR rehabilitation systems utilized in the included studies consist of a server computer with a web camera and an optical see-through HMD connected to a personal computer [24, 25, 31–37, 39]. In these systems, patients followed the displayed instruction and performed the corresponding movement. In the meantime, the computer sensed the patients' movement and sent the information to the HMD in order to repeat the task or move to the next level. However, due to the inherent limitations of the HMD devices, unexpected physical side effects (e.g., fatigue and nausea) still cannot be completely avoided. Researchers have already started to look for alternatives. The rest of the included studies developed the 3D interactive augmented reality system using the motion-tracking Kinect sensor (Microsoft Inc., Redmond, WA, USA) [26–30, 38]. A 3D depth map was created by the sensor, and the patients in front of the sensor can be detected as 3D objects on a computer. Patients interacted with the virtual objects on the screen and watch their movement (e.g., gait and posture) at the same time.

### 3.3. AR Intervention for Lower Limb Rehabilitation of Elderly Adults

The first group of studies investigated the effects of AR interventions for lower limb rehabilitation of healthy elderly adults. Yoo et al. [24] first started AR interventions on elderly women, intending to investigate the effects of AR-based Otago exercise on balance, gait, and fall efficacy. Subjects were asked to perform a 60-minute Otago exercise with or without the AR environment 3 sessions per week for 12 weeks in total. The Otago exercise consists of lower limb muscle strengthening exercises and balance training. The results showed that AR-based Otago exercise significantly improved subjects' lower limb balance, gait velocity, cadence, step length, and stride length, while reduced the fall risk. Similarly, Lee et al. [25] employed the same AR intervention protocol on elderly women. What is more, they further compared the AR-based Otago exercise with yoga or self-exercise programs, and the effects of these interventions on lower limb muscle strength were further investigated. Similar results were found in terms of balance and gait functions, and Lee et al. [25] also confirmed the significant effects of AR-based Otago exercise on knee flexion and ankle dorsiflexion strength.

Two subsequent studies determined the effects of a 3D interactive AR program on the balance and mobility rehabilitation of elderly adults. Im et al. [26] conducted a before-after study, and they required subjects to perform the 30-minute three-dimensional interactive AR program for 10 sessions in 12 weeks. Several tasks that enable specific motions of specific lower limb joints were designed in this program. Specifically, the balloon game for the hip joint, the cave game for the knee joint, and the rhythm game focuses on one-leg standing ability. Both the lower limb balance and mobility were improved after the training, and the success rate and response time for each game also improved gradually across sessions. In Ku et al. [27] study, subjects were randomly divided into two groups, and the control group was asked to perform the 30-minute conventional physical fitness program 3 times per week for 1 month, while the experimental group performed the same 3D interactive AR program 3 times per week for 4 weeks. However, their results only confirmed that the 3D interactive AR program can enhance the balance ability more effectively than the conventional physical fitness program, and they speculated that it is highly associated with motor learning mechanism as the subjects had to make the movement according to the contents in AR environment.

The last three studies were all published in 2020, and they all provided positive results in terms of the effects of AR-based intervention on lower limb rehabilitation of elderly adults. Chen et al. [28] investigated the acute one-time effect of AR-based cognitive-motor intervention training on fall risk of the elderly. Three specific training programs were performed, including the wall dodging game, the fruit picking game, and the rats stomping game. Their results indicated that the AR-based exergame system could help to reduce the fall risk of the elderly in the long run. Jeon and Kim [29] compared the effects of an AR-based muscle reduction prevention exercise program with a control program on muscle parameters, physical performance, and exercise self-efficacy of elderly women. Subjects in the experimental group were required to perform a 30-minute AR-based aerobic and flexibility exercise 5 times a week for 12 weeks, while the exercise for the control group was not specified. They found that the AR-based exercise program is more effective in preventing muscle reduction, improving physical performance, and inducing physical activity in elderly women. The last study conducted by Chen et al. [30] is aimed at determining whether AR-assisted training with selected Tai Chi movements could be as effective as the complete traditional Tai Chi movements in increasing lower limb muscle strength and enhancing balance control. Subjects were asked to perform the selected Tai Chi movements using the AR training system or complete the 24-form Yang-style Tai Chi 30 minutes per time with 3 sessions per week for 8 weeks. The results confirmed their hypothesis that AR-assisted training with selected Tai Chi movements could be at least as effective as the complete sequence for improving muscle strength and balance control. In conclusion, all studies have confirmed the benefit of AR intervention for lower limb rehabilitation of healthy elderly adults, with favorable results found in lower limb balance, muscle strength, gait, physical performance, and fall efficacy. However, whether AR intervention could achieve greater effects on lower limb rehabilitation of healthy elderly adults when compared to the same training protocol without AR requires further investigation.

### 3.4. AR Intervention for Lower Limb Rehabilitation of Stroke Patients

The second set of identified studies focused on the effects of AR intervention for lower limb rehabilitation of stroke patients. The first research was performed to compare the effects of an obstacle training program with or without an AR environment on gait parameters of stroke patients [31]. Subjects completed six intervention sessions in 2 weeks in which they were asked to step over the virtual obstacle or real foam objects during a 60-minute walking training. The results found that the virtual obstacle walking training showed greater improvement in fast walk velocity, but both training methods exhibited similar effectiveness in self-selected walk velocity, stride length, and walking endurance. The following two studies employed similar AR-based interventions on stroke patients [32, 33]. The functional electrical stimulation was conducted by a functional electrical stimulator which was attached to the proximal and distal part of the tibialis anterior muscle when subjects were asked to perform ankle dorsiflexion or treadmill walking with or without an AR environment. Although the training set is slightly different, both studies found that AR-based functional electrical stimulation was more effective in improving lower limb muscle strength of stroke patients, but Kim and Lee [33] further demonstrated that functional electrical stimulation with and without AR exhibited the same improvement in balance and gait function. Lee et al. [34] and Park et al. [35] also employed similar AR-based interventions on stroke patients. Subjects of the experimental group were asked to further perform the 30-minute AR-based postural control training after the general physical therapy 3 sessions per week for 4 weeks. The AR-based training program incorporated three stages with different body positions (i.e., lying position for stage 1, sitting position for stage 2, and standing position for stage 3). The results of these two studies both demonstrated that AR-based postural control training has greater effects on gait function while no significant difference in balance between groups. The last paper conducted in 2020 is a case report focused on the effects of an AR-based parkour course on the gait function of a stroke patient with chronic minor gait impairment [36]. The subject was required to overstep obstacles during the parkour course. Their results found that the patient changed his gait pattern during the AR-based parkour course compared to the clinical gait assessments, which indicated that the AR-based intervention has the potential to provide gait rehabilitation for stroke patients. To summarize, in patients who had a stroke, AR intervention could help to improve their lower limb balance, muscle strength, and gait. However, similar to the findings of AR intervention on healthy elderly adults, the significant effects of AR training compared to non-AR one need further verification.

### 3.5. AR Intervention for Lower Limb Rehabilitation of Parkinson Patients

The remaining three studies all investigated the effects of AR-based interventions on gait functions of Parkinson patients. Espay et al. [37] investigated the effects of at-home walking training with a closed-loop AR cueing device on the gait function of Parkinson patients, and they found that the 30-minute training twice daily for 2 weeks enhanced walking velocity and stride length. Palacios-Navarro et al. [38] aimed to determine the effects of an AR-based mole stomping game on the gait function of Parkinson patients, and they also found that the 30-minute game with 4 sessions per week for 5 weeks is effective to improve the completion time score and walk function. However, some conflicting and equivocal results have been proposed by Janssen et al. [39]. In their study, the acute effects of AR-based visual cues on freezing of gait and turning in place of Parkinson patients were assessed, and the results showed that the AR-based visual cues did not reduce freezing of gait and even worsen some gait kinematics and turning in place. They speculated that the insufficient AR-based visual cues, influences of smart glasses, and subjects' unfamiliarity with the training could all be associated with the detrimental effects. According to the results obtained, the benefit of AR intervention for gait function of Parkinson patients is still conflicting, and more studies in this field are warranted.

## 4. Discussion

This systematic review summarized and analyzed previous studies that explored the effects of AR-based interventions on lower limb rehabilitation, with the aim to determine whether it could contribute significant benefits to the larger population and further reveal its potential applications to further enhance lower limb rehabilitation.

According to the results of this study, the significant effects of AR-based interventions on lower limb rehabilitation have been initially confirmed. To be specific, the AR-based interventions have currently been conducted for elderly adults, stroke patients, and Parkinson patients. Favorable results were achieved in dynamic balance, gait spatiotemporal variables, gait kinematics, muscle mass, muscle activation, muscle force, physical performance, and fall efficacy. Nevertheless, one study that investigated the effects of an AR-based system on gait function and turning in place of Parkinson patients did not come out with any positive results when compared to the preintervention; they demonstrated that the insufficient cues, influences of AR glasses, and subjects' unfamiliarity with the training could be the main reasons for this controversy [39]. In addition, it is worth mentioning that some studies obtained no significant differences in lower limb rehabilitation after AR treatments when compared to the same interventions only without AR or conventional training programs [27, 30, 33]. In other words, interventions with or without AR seem to provide similar rehabilitation benefits. Chen et al. [30] investigated the effects of AR-assisted training with selected Tai Chi movements on lower limb muscle strength and balance control, and their results found that AR-assisted training with selected Tai Chi movements achieved similar effects with the complete sequence. Ku et al. [27] investigated the effects of a 3D interactive AR program on balance and gait function of the elderly, while only balance was found significant when compared to the conventional physical fitness program, and they speculated that the balance improvement is only because of motor learning mechanism. Overall, this review adds support to previous studies indicating that patients could benefit from AR-based rehabilitation intervention, at least the same as the conventional program. However, given the small sample size included in these studies, more research with a larger sample size is much warranted for further verification.

There is great variability in AR-based training programs evaluated in these included studies, which on one hand makes it hard to determine a general intervention that could contribute benefits to the larger population, while on the other hand, it is supported that AR can provide the opportunities to extend beyond rote rehabilitation training by adding more exercises that is highly related to daily living. Based on the needs and actual motor functions of the patients, an appropriate AR intervention mode could be further designed [18]. In terms of the intervention time setting, it ranged from only one session to 5 sessions per week for 12 weeks, while a thorough examination of these included trials found that 30 or 60 min per session at 3 to 5 times per week for a total of 8 to 12 weeks was the most frequently used setting. The intensity and duration of AR training can be further modified based on the patients' motor condition during the rehabilitation process [18]. Nevertheless, the diverse AR treatments may indicate that this technology is still in the early stage of clinical application, and some drawbacks of AR intervention should be resolved to promote better rehabilitation outcomes. Firstly, although the wearable AR device has a strong sense of immersion and can bring real-time interaction, the induced side effects during and after the intervention (i.e., nausea and fatigue) may reduce the enthusiasm of patients for training. Moreover, some technological or user interface shortcomings may also limit its clinical applications. For example, it is currently impossible to apply the AR system in an unprepared environment since this technology relies on tracking methods in the prepared environment [19].

Two potential limitations that existed should be noted here. Firstly, it is in some cases difficult to compare these findings statistically such as performing a meta-analysis since the homogeneity of instruments, measurement scales, and units applied in these included studies was relatively limited [40, 41]. Moreover, there are limited numbers of studies that were available, while it becomes much fewer after being divided into different categories by the types of participants, which might impact the integration of the results.

## 5. Conclusions

Based on the results of this literature review, it was found that AR-based interventions have been applied for the lower limb rehabilitation of balance, gait, muscle, physical performance, and fall efficacy of the elderly, stroke, and Parkinson patients. Favorable results were achieved at least the same as the interventions without AR except for the turning and timing in the freezing of gait of Parkinson patients. However, given the infancy of this technology in clinical practices, more robust trials with larger sample sizes and greater homogeneity in terms of devices and treatment settings are warranted for further verification. On the other hand, it is proposed that the future development of AR systems should focus on the following several aspects to make it widespread in the motor rehabilitation field. First, some high technologies such as artificial intelligence should be integrated into the AR rehabilitation systems as they can accurately track patients' progress and intelligently adapt the training programs based on their feedback. Moreover, the development of an AR-based system on mobile devices could contribute to more benefits because it can realize the remote monitoring of patients' recovery and provide real-time attention with lower costs. Finally, more game-based rehabilitation content targeted at different populations would also be of interest for AR systems as it may further improve the users' motivation.

## Figures and Tables

**Figure 1:** The review flow chart.

**Table 1:** The basic characteristics of the included studies.

Reference	Objective	Participant	Intervention	Intervention frequency	Outcome test
AR intervention for lower limb rehabilitation of elderly adults					
Chen et al. [30]	Investigated the effects of AR-assisted training with selected Tai Chi movements on balance and muscle strength of older adults.	Elderly men (*N* = 28) Experimental group (*N* = 14, age, 72.2 ± 2.8 years) Control group (*N* = 14, age, 75.1 ± 5.5 years)	Experimental group: AR-assisted training with selected Tai Chi movements Control group: 24-form Yang-style Tai Chi movements	30 min per time with 3 sessions per week for 8 weeks	Balance: Berg balance scale test, timed up and go test, functional reach test Muscle strength: lower limb muscle strength test
Yoo et al. [24]	Investigated the effects of AR-based Otago exercise on balance, gait, and fall efficacy of older adults.	Elderly women (*N* = 21) Experimental group (*N* = 10, age, 72.90 ± 3.41 years) Control group (*N* = 11, age, 75.64 ± 5.57 years)	Experimental group: AR-based Otago exercise for muscle strengthening and balance training Control group: Otago exercise for muscle strengthening and balance training	60 minutes per time with 3 sessions per week for 12 weeks	Balance: Berg balance scale test Gait: velocity, cadence, step length, and stride length Fall: fall efficacy test
Lee et al. [25]	Investigated the effects of AR-based Otago exercise on balance, muscle strength, and physical factors in falls of older adults.	Elderly women (*N* = 30) Experimental group (*N* = 10, age, 72.60 ± 2.67 years) Control group 1 (*N* = 10, age, 75.80 ± 5.47 years) Control group 2 (*N* = 10, age, 76.40 ± 5.54 years)	Experimental group: AR-based Otago exercise for muscle strengthening and balance training Control group 1: yoga Control group 2: elastic band exercise program	60 minutes per time with 3 sessions per week for 12 weeks	Balance: foot print test Muscle strength: lower limb muscle strength test Fall: short Morse fall scale test
Im et al. [26]	Investigated the effects of 3D interactive AR system on balance and kinematic function of older adults.	Elderly adults (*N* = 18, age, 64.72 ± 7.27 years)	3D interactive AR system	30 minutes per time for 10 sessions in 12 weeks	Balance: Berg balance scale test; timed up and go test Gait: hip and knee joint angle
Jeon and Kim [29]	Investigated the effects of AR-based muscle reduction prevention exercise program on muscle parameters, physical performance, and exercise self-efficacy of older adults.	Elderly women (*N* = 27) Experimental group (*N* = 13, 72.77 ± 3.79 years) Control group (*N* = 14, 72.71 ± 3.64 years)	Experimental group: AR-based muscle reduction prevention exercise program Control group: NA	30 minutes per time with 5 sessions per week for 12 weeks	Muscle mass: bioelectrical impedance analysis Muscle function: gait speed and hand grip strength Physical performance: senior fitness test Exercise self-efficacy: exercise self-efficacy scale
Chen et al. [28]	Investigated the effects of AR-based exergame system on fall risk of older adults.	Elderly adults (*N* = 25, age, 71.48 ± 4.09 years)	AR-based exergame system	One time	User experience: user experience questionnaire
Ku et al. [27]	Investigated the effects of 3D interactive AR system on the balance and mobility of older adults.	Elderly adults (*N* = 36) Experimental group (*N* = 18, 64.7 ± 7.27 years) Control group (*N* = 18, 65.0 ± 4.77 years)	Experimental group: 3D interactive AR system training Control group: conventional physical fitness program	Conventional physical fitness program: 30 min per time with 3 sessions per week for 1 month 3D interactive AR system training: 30 min per time with 3 sessions per week for 4 weeks	Balance and mobility: lower-extremity clinical scale scores, fall index, automatic balance score
AR intervention for lower limb rehabilitation of stroke patients					
Lee et al. [34]	Investigated the effects of AR-based postural control training on balance and gait function of stroke patients.	Stroke patients (*N* = 21) Experimental group (*N* = 10, age, 47.9 ± 12.0 years) Control group (*N* = 11, age, 54.0 ± 11.9 years)	Experimental group: AR-based postural control training+ general physical therapy program Control group: general physical therapy program	General physical therapy program: 30 minutes per time with 5 sessions per week for 4 weeks Additional AR-based postural control training: 30 minutes per time with 3 sessions per week for 4 weeks	Balance: Berg balance scale test, timed up and go test Gait: velocity, cadence, step length, and stride length
Park et al. [35]	Investigated the effects of AR-based postural control training on balance and gait function of stroke patients.	Stroke patients (*N* = 20) Experimental group (*N* = 10, 47.38 ± 13.44 years) Control group (*N* = 10, 53.50 ± 12.43 years)	Experimental group: AR-based postural control training+ conventional physical therapy Control group: conventional physical therapy	Conventional physical therapy: 60 minutes per time with 5 sessions per week for 4 weeks Additional AR-based postural control training: 30 minutes per time with 3 sessions per week for 4 weeks	Balance: Berg balance scale test Gait: 10-meter walk test
Kim et al. [33]	Investigated the effects of AR-based functional electrical stimulation during treadmill gait training on balance, gait, sand muscle trength of stroke patients.	Stroke patients (*N* = 28) Experimental group (*N* = 9, age, 47.44 ± 8.39 years) Control group 1 (*N* = 10, age, 51.50 ± 12.90 years) Control group 2 (*N* = 9, age, 49.11 ± 11.02 years)	Experimental group: AR-based functional electrical stimulation during treadmill gait training Control group 1: functional electrical stimulation during treadmill gait training Control group 2: treadmill gait training	20 minutes per time with 3 sessions per week for 8 weeks	Balance: Berg balance scale test Gait: timed up and go test Muscle strength: lower limb muscle strength test
Jung et al. [32]	Investigated the effects of AR-based EMG-triggered functional electric simulation on the range of motion, muscle activation, and muscle strength of ankle joint of stroke patients.	Stroke patients (*N* = 10) Experimental group (*N* = 5, age, 58.40 ± 8.26 years) Control group (*N* = 5, age, 57.80 ± 10.23 years)	Experimental group: AR-based EMG-triggered functional electric simulation Control group: EMG-triggered functional electric simulation	20 minutes per time with 5 sessions per week for 4 weeks	Muscle activation (ankle) Muscle strength (ankle) Ankle range of motion
Jaffe et al. [31]	Investigated the effects of AR-based walking program on the walking function of patients with poststroke hemiplegia.	Stroke patients (*N* = 20, age, 60.7 ± 2.3 years)	AR-based obstacle training program Obstacle training program	60 minutes per time with 6 sessions for 2 weeks	Gait: gait velocity, step length, ability to step over obstacles, and walking endurance
Held et al. [36]	Investigated the effects of AR for gait impairment after stroke system on overground walking function of a stroke patient.	Stroke patient (*N* = 1, age, 74 years)	Experimental group: AR for gait impairment after stroke system Control group: clinical gait assessments	One time	Gait: hip, knee, and ankle joint angle, position of the center of mass
AR intervention for lower limb rehabilitation of Parkinson patients					
Espay et al. [37]	Investigated the effects of at-home training with a closed-loop AR cueing device on the walking function of Parkinson patients.	Parkinson patients (*N* = 13, age, 73.3 ± 11.7 years)	At-home training with closed-loop AR cueing device	30 minutes per timetwice daily for 2 weeks	Gait: gait velocity, stride length, cadence, and freezing of gait questionnaire
Janssen et al. [39]	Investigated the effects of AR visual cues on freezing of gait and turning in place of Parkinson patients experiencing freezing of gait.	Parkinson patients (*N* = 16, age, median 69 years)	AR visual cues	One time	Freezing of gait: percent time frozen, number, and duration Axial kinematics: medial COM deviation and head-pelvis separation Gait: cadence, step height, and stride time
Palacios-Navarro et al. [38]	Investigated the effects of AR-based rehabilitation games on the walking function of Parkinson patients.	Parkinson patients (*N* = 7, age, 67 ± 3 years)	AR-based rehabilitation games	30 min per time with 4 sessions per week for 5 weeks	Gait: 10-meter walk test score

Note: AR: augmented reality; COM: center of mass; NA: not available.

## Data Availability

The data used to support the findings of this study are included within the article.
